RETRACTED

# Causal Relationship Between Diet, Lipids, Immune Cells, and Chronic Fatigue Syndrome: A Two‐Mediation Mendelian Randomization Study

**DOI:** 10.1002/fsn3.70424

**Published:** 2025-06-22

**Authors:** Jixu Li, Qi Qin, Yiran Zhu, Yulu Qian, Jialu Yin, Xin Gao, Huijuan Wen, Pei Wang

**Affiliations:** ^1^ Department of Cardiology Affiliated Hospital of Nanjing University of Chinese Medicine Nanjing China; ^2^ Affiliated Hospital of Nanjing University of Chinese Medicine Nanjing China; ^3^ Department of Gastroenterology The First Clinical College of Shandong University of Traditional Chinese Medicine Jinan China; ^4^ Department of Geriatrics, Nanjing First Hospital Nanjing Medical University Nanjing China

**Keywords:** chronic fatigue syndrome, diet, immune cells, lipids, mediation, Mendelian randomization

## Abstract

Chronic fatigue syndrome (CFS) is a disorder characterized by severe unexplained fatigue and is associated with various factors including infections, immune responses, genetics, and environmental influences. However, the underlying mechanisms and possible interventions for CFS remain unclear. We used a two‐mediated MR method to investigate causal relationships between diet, lipid levels, immune cells, and CFS. Our findings suggest that certain lipids, specifically low‐density cholesterol, apolipoprotein E, and apolipoprotein B, contribute to CFS development. Conversely, high‐density lipoprotein cholesterol and apolipoprotein A1 may delay the onset of the syndrome. Additionally, we explored how lipids affect fatigue through immune cell mediation. Factors, such as hematopoietic stem cell absolute count, the percentage of CD3‐natural killer lymphocytes, and IgD presence on IgD+ CD38+ B cells may mediate the causal pathway linking lipids to CFS. Furthermore, we examined the relationship between diet, lipids, and CFS. This indicated that specific dietary selections, like alcohol intake, a preference for chili peppers, and an affinity for breakfast, contributed to CFS. Conversely, cheese and pork consumption were protective factors against CFS. The protective effect of cheese consumption on CFS was mediated by apolipoprotein A1 and high‐density lipoprotein cholesterol. In conclusion, the study established an ecological chain: cheese consumption leads to increased high‐density lipoprotein cholesterol and alters immune cell phenotypes—specifically, increasing the percentage of CD3‐lymphocytes and IgD on IgD+ CD38+ B cells—ultimately influencing the development of CFS. These findings enhance our understanding of how lipid levels and immune factors are related to CFS and how dietary choices can potentially mitigate the syndrome.

## 1 Introduction

CFS is predominantly defined by fatigue as its principal symptom. In addition, it involves multiple pathophysiological changes across various systems, including alterations involving the immune microenvironment, metabolic abnormalities, microbiota dysregulation, central nervous system disorders, and circulatory issues. These factors can influence the onset and progression of CFS (Apostolou and Rosén 2024; Holden et al. 2020; Morris et al. 2022). Several prospective studies have confirmed links between dyslipidemia and immunoinflammatory abnormalities and the incidence of CFS (Mahemuti et al. 2023; Nkiliza et al. 2021). Recent lipidomic studies have identified specific dyslipidemia associated with CFS, including irregularities involving phospholipids, sphingomyelins, cholesteryl esters, total cholesterol (TC), and triglyceride (TG) levels (Germain et al. 2020, 2018). These lipid profiles may serve as unique biomarkers for the diagnosis of CFS, associated with perturbations in immune, inflammatory, and metabolic processes. This provides a new theoretical foundation for understanding the pathophysiology of CFS (Brenu et al. 2011). Patients with CFS often exhibit decreased natural killer (NK) cell levels, alongside increased levels of circulating CD4+ and CD8+ T cells, T regulatory cells, and memory B cells (Brenu et al. 2014). Brenu's research indicates that impaired NK cell lysis, together with elevated antibodies against KIR3DL1 and cytokines associated with cytotoxicity, may lead to decreased NK cytotoxicity, which is closely associated with the development of CFS (Brenu et al. 2013). Furthermore, immune cells, such as NK cells, T cells, and macrophages require lipids for energy and produce lipid mediators that activate and regulate inflammatory responses (Brenu et al. 2014). By regulating lipoprotein metabolism during inflammatory states, the body alters plasma lipoprotein concentrations, impacting levels of TC and TG. Abnormal lipid levels may promote inflammation (Hornig et al. 2015). For example, arachidonic acid—an omega‐6 polyunsaturated fatty acid—can be oxidized via enzymatic reactions to mediate inflammatory responses (Marklund et al. 2019). In conclusion, lipids are bi‐directionally linked to immuno‐inflammation, and the interplay between these two factors influences the development of CFS.

RETRACTED

CFS is a long‐term condition with no clear etiology and limited treatment options. Patients can improve their prognosis by modifying their daily lifestyle. Research has shown that dietary interventions can positively affect lipid metabolism and alleviate fatigue. By implementing scientific dietary modifications and receiving nutritional education, patients' quality of life and overall health can be enhanced. Studies have highlighted that consuming foods rich in coenzyme Q10, such as pork liver, beef, and corn, can significantly reduce cognitive fatigue and overall feelings of fatigue. Additionally, foods rich in omega‐3 fatty acids, such as sardines, salmon, and flaxseed oil, can lower TG levels and boost high‐density lipoprotein cholesterol (HDL‐C) levels (Castro‐Marrero et al. 2021; Chen et al. 2019). In summary, enhancing lipid metabolism through dietary changes affects multiple mechanisms, including immunity and inflammation, thereby slowing the progression of CFS.

Emerging epidemiological research has highlighted a link between lipids and CFS, suggesting that dietary changes may help alleviate this condition. However, the precise mechanism remains unclear, and many studies had limited sample sizes, indicating the need for more robust multicenter randomized controlled trials (Weigel et al. 2021; Zerón‐Rugerio et al. 2024). Genome‐wide association studies (GWAS) have tremendous potential to shed light on the susceptibility to complex traits and to develop genetic tools to explore intricate associations in this area. This is particularly relevant in terms of the relationships among lipids, CFS, and diet. By leveraging genetic information, we can better address challenges, such as reverse causation, and confounding bias (Ellervik et al. 2021). While previous MR studies have utilized various methodologies, our current research takes a new approach by employing dual‐mediated MR for the first time (He et al. 2023; Jiang et al. 2024). We aimed to investigate the causal link between blood lipids and CFS, focusing on immune cells as mediators. In addition, we examined how dietary habits may positively affect CFS, using blood lipids as a key factor. Ultimately, this study provides valuable, evidence‐based insights into the pathogenesis, prevention, and treatment of CFS, paving the way for informed medical advances.

## 2 Methods

This study was conducted in accordance with the STROBE‐MR declaration for enhanced epidemiological observational studies and followed the recommended checklist (Skrivankova et al. 2021).

### 2.1 Research Design

We used publicly available GWAS data to conduct a dual‐mediated MR study. Therefore, we investigated the influence of different dietary approaches and lipid levels on CFS development. Moreover, we used a two‐step MR method to understand how lipids and immune cells might mediate their effects under these conditions (Figure 1).

**FIGURE 1:** The causal relationship between diet, lipids, immune cells, and CFS was investigated using a dual‐mediated Mendelian randomization method. The causal exposure relationship between blood lipids and CFS was first investigated using immune cells as a mediator (green color *β*0, *β*1, *β*2); then the ameliorative effect of dietary consumption on CFS was explored using blood lipids as a mediator (blue color *β*0, *β*1, *β*2).

RETRACTED

### 2.2 Data Sources

In this research, we explored the GWAS data for CFS, which was carefully sourced from the IEU GWAS database. This impressive dataset included insights from 7363 samples and featured 163,803,05 SNPs, providing a robust foundation for our findings. We also examined lipid data, which comprised eight essential exposure factors. We gathered GWAS data on important biomarkers, such as TC, TG, HDL‐C, low‐density lipoprotein cholesterol (LDL_C), lipoprotein A (Lp (a)), and apolipoprotein B (Apo B) from the UK Biobank (UKB). Additionally, we complemented our analysis with collated and summarized data from the IEU database, as well as data for apolipoprotein A1 (Apo A1) and apolipoprotein E (Apo E) from the same reliable platform.

Regarding dietary patterns, our study involved a detailed examination of 38 dietary consumption and 187 dietary preferences. Among these factors, we considered a variety of food items, including beef consumption, decaffeinated coffee consumption, dried fruit consumption, ground coffee consumption, percentage fat in milk consumption, and so on. We also explored dietary preferences that capture individual likes, such as alcohol liking, apple juice liking, bitter ale liking, fruit juice liking, lager liking, f‐seafood liking, and so on. We leveraged GWAS summary data from the UKB for a comprehensive analysis. Immune cell GWAS phenotypes were meticulously gathered from the GWAS database, which allowed us to download a broad spectrum of immune phenotypes (No. GCST90001391 to GCST90002121). This encompassed vital metrics, such as the percentages of specific B cells and dendritic cells and counts of various T cell types, including active and resting CD4 regulatory T cells, along with a total of 731 other immune cell phenotypes. All datasets utilized in our study are publicly available (Table S1).

### 2.3 Selection of Instrumental Variables

The MR study is a statistical approach grounded in Mendelian inheritance principles, highlighting how parental alleles are randomly distributed to their offspring. This innovative study design explored causal links between exposures and their outcomes, providing valuable insights. It operates based on three fundamental principles: (1) Genetic variants serving as instrumental variables (IVs) should have a strong relationship with dietary patterns and lipid levels. (2) These variables should not be affected by confounding factors. (3) IVs must influence CFS solely through dietary patterns and lipid levels not through other factors (Davies et al. 2018).

RETRACTED

In selecting IVs, we adhered to three fundamental assumptions. Several additional steps were implemented to enhance the accuracy and reliability of the analysis. (1) Lipids and dietary style were used as exposure factors, and SNPs with significance to both (*p* < 5 × 10^−6^) were extracted as IVs, with CFS as the outcome variable. (2) The linkage disequilibrium parameter *r* ^2^ threshold was set to 0.001, and the genetic distance was set to 10,000 kb. (3) The data were preprocessed such that the effect alleles of the IVs were aligned, that is, SNPs identified in the exposure GWAS were coordinated with SNPs in the outcome GWAS, and the alleles were aligned on the same strand to ensure base pair identity between exposure and outcome GWAS. (4) The *F* statistic was calculated for all SNPs in the analysis, with *F* > 10 indicating the absence of weak IV bias (Sekula et al. 2016).

### 2.4 MR Analysis

This study employed four methods for MR analysis: inverse variance weighted (IVW), MR Egger, weighted median (WME), and weighted mode. The IVW method took center stage in our primary analysis because of its outstanding capability to estimate causal effects within MR studies (Brown and Knowles 2021). By aggregating MR effect estimates from individual SNPs, the IVW method enables us to calculate a comprehensive weighted estimate of potential causal effects. The results of the IVW analyses are most reliable when the IVs do not suffer from level multinomial and if *p* < 0.05, which indicates the presence of heterogeneity. In such cases, a random effects model was used for causal effect estimation. Otherwise, a fixed effects model was used.

A mediator is considered to be present if the following conditions are met: (1) The exposure factor was associated with the study outcome without adjusting for the mediator (*β*0). (2) There was a correlation between the exposure factor and the mediator (*β*1). (3) There was a correlation between the mediator and the study outcome (*β*2). The mediator ratio was calculated as (*β*1*β2/*β*0) (Carter et al. 2021).

### 2.5 Sensitivity Analysis

To assess heterogeneity among individual genetic variants and to evaluate potential violations of the MR assumptions, we conducted a series of statistical methods and sensitivity analyses. (1) Cochran's *Q* test: For *p* < 0.05, the Cochran's *Q* test indicated the presence of heterogeneity, and the causal effects were estimated using a random effects model; otherwise, a fixed effects model was used (Kulinskaya et al. 2020). (2) Egger's intercept method was used to check for horizontal heterogeneity, that is, whether the selected instrumental variable significantly affected the outcome variable through a pathway other than exposure. If *p* < 0.05 for the Egger intercept, it indicates the presence of horizontal pleiotropy, violating the assumption of independence and the assumption of exclusivity; conversely, it indicates that the exposure does not significantly affect the outcome variable through unintended pathways (Cho et al. 2020). (3) MR‐PRESSO test: The MR‐PRESSO method is used to identify and correct for outliers, and by setting the number of distributions to 10,000, MR‐PRESSO can efficiently identify and deal with outliers (Cho et al. 2020). (4) Leave‐one‐out sensitivity analysis: The leave‐one‐out sensitivity test assesses the effect of each SNP on the overall MR analysis results by excluding them one by one (Ye et al. 2024). (5) Funnel plot symmetry checks: The stability and reliability of the results of MR analyses can be further checked by observing the symmetry of funnel plots (Sekula et al. 2016).

RETRACTED

### 2.6 Statistical Processing

All statistical analyses were conducted using R v.4.3.0 and the software packages “TwoSampleMR” and “Mendelian Randomization”. Two‐sided tests were performed with a significance level of *α* = 0.05.

## 3 Results

### 3.1 Relationship Between Lipid Levels and CFS

Univariate MR analysis of the IVW method showed that TC (IVW, OR: 1.1, 95% CI: 1.02–1.19, *p* = 0.016), LDL‐C (IVW, OR: 1.12, 95% CI: 1.02–1.22, *p* = 0.017), apo B (IVW, OR: 1.07, 95% CI: 1.01–1.14, *p* = 0.019), and apo E (IVW, OR: 1.12, 95% CI: 1–1.24, *p* = 0.042) were all significantly associated with an increased risk of CFS. HDL‐C (IVW, OR: 0.92, 95% CI: 0.86–1, *p* = 0.038) and apo A1 (IVW, OR: 0.9, 95% CI: 0.82–0.99, *p* = 0.032) were significantly and negatively correlated with the risk of CFS. Meanwhile, TG (IVW, OR: 0.94, 95% CI: 0.87–1.02, *p* = 0.135) and lp(a) (IVW, OR: 0.96, 95% CI 0.89–1.03, *p* = 0.281) were not causally associated with the onset of CFS (Figures 2 and 3).

**FIGURE 2:** Causal relationship between different types of lipids and CFS. SNPs: number of SNPs. CI, confidence interval; OR, ratio of ratios.

**FIGURE 3:** Funnel and scatter plots of the causal estimates of different types of lipids on fatigue syndrome. (A–H) funnel plots; (I–P) scatter plots. (A and I) TC on CFS. (B and J) TG on CFS. (C and K) HDL‐C on CFS. (D and L) LDL‐C on CFS. (E and M) Apo A1 on CFS. (F and N) Apo E on CFS. (G and O) Lp (a) on CFS. (H and P) Apo B on CFS.

### 3.2 Relationship Between Immune Cells and CFS

Two‐sample MR analysis used 731 immune cell phenotypes as exposure factors and CFS as the outcome variable. The analysis identified 35 immune cell phenotypes that are causally associated with CFS based on the IVW method. Among these were 19 types of lymphocytes, two types of monocytes, two types of granulocytes, and 1 type of hematopoietic stem cell. Further analysis revealed that 22 immune cell phenotypes were positively associated with an increased risk of developing CFS, with CD4+/CD8+ T cells showing the most significant association (IVW, OR: 1.14, 95% CI: 1.05–1.25, *p* = 0.002). In contrast, 13 immune cell phenotypes were protective against CFS. This indicates that a higher level of these protective immune cell phenotypes is negatively correlated with the risk of disease development. Notably, there was a pronounced negative correlation for CD28+ CD4− CD8‐T cells (IVW, OR: 0.85, 95% CI: 0.76–0.95, *p* = 0.004) (Figure 4).

RETRACTED

**FIGURE 4:** Causal relationship between different types of immune cell phenotypes and CFS.

### 3.3 Results of Immune Cell Phenotype Mediation Effect Analysis

Mediation analysis of immune cells was conducted to determine whether they mediated the effects of lipids on CFS. Using two‐step MR analysis, this study identified three immune cell characteristics that could mediate the causal relationship between lipids and CFS: hematopoietic stem cell absolute count, the percentage of NK CD3− lymphocytes, and IgD on IgD+ CD38+ B cells. The results from the two‐step mediation analysis revealed a direct effect size of −0.080 for the impact of HDL‐C on CFS. Specifically, the mediated effect sizes for the identified immune cell characteristics were − 0.010 for hematopoietic stem cell absolute count, −0.004 for NK% CD3− lymphocytes, and −0.005 for IgD on IgD+ CD38+ B cells. These corresponded to mediated effect ratios of 12.6%, 4.9%, and 6.7%, respectively (Table 1).

**TABLE 1:** Intermediate MR analysis.

Exposure	Meditation	Outcome	*β*1 effect	*β*2 effect	Indirect effect	Direct effect	Total effect	Mediation effect
HDL_C	Hematopoietic stem cell absolute count	CFS	−0.203	0.050	−0.010	−0.080	−0.070	0.126
HDL_C	Natural Killer %CD3− lymphocyte	CFS	0.142	−0.0281	−0.004	−0.080	−0.076	0.049
HDL_C	IgD on IgD+ CD38+ B cell	CFS	−0.127	0.042	−0.005	−0.0804	−0.075	0.067
Cheese consumption	Apolipoprotein A1	CFS	0.732	−0.101	−0.074	−1.730	−1.656	0.043
Cheese consumption	High‐density lipoprotein cholesterol	CFS	1.072	−0.080	−0.086	−1.730	−1.644	0.050

### 3.4 Association of Genetically Predicted Dietary Styles With CFS

Among the 38 dietary consumptions and 187 dietary likes investigated within various dietary styles, several factors were found to influence the development of CFS. Alcohol consumption was identified as a detrimental factor, with an OR of 1.56 (95% CI: 1.19–2.04, *p* = 0.001). Additionally, the consumption of champagne or white wine had an OR of 4.29 (95% CI: 1.20–15.35, *p* = 0.025), and spirits consumption showed a significantly higher risk with an OR of 13.7 (95% CI: 3.19–58.87, *p* = 0.0004). Cooked vegetable consumption also presented a higher risk, with an OR of 3.78 (95% CI: 1.14–23, *p* = 0.049), which was matched by the number of individuals consuming vegetables. Other detrimental factors included a preference for chili peppers (OR: 1.11, 95% CI: 1.01–1.22, *p* = 0.035) and liking for pizza (OR: 1.25, 95% CI: 1.02–1.54, *p* = 0.034). In contrast, certain dietary factors appear to protect against CFS. Cheese consumption was associated with an OR of 0.18 (95% CI: 0.04–0.86, *p* = 0.032), and pork intake showed an even stronger protective effect with an OR of 0.12 (95% CI: 0.02–0.62, *p* = 0.012) (Figures 5 and 6).

RETRACTED

**FIGURE 5:** Causal relationship between different types of immune cell phenotypes and CFS. SNPs: number of SNPs. CI, confidence interval; OR, ratio of ratios.

**FIGURE 6:** Funnel and scatter plots of the causal estimates of different types of diets on CFS. (A–H) funnel plots; (I–P) scatter plots. (A and I) Alcohol consumption on CFS. (B and J) Champagne or white wine consumption on CFS. (C and K) Cheese consumption on CFS. (D and L) Cooked vegetables consumption on CFS. (E and M) Pork consumption on CFS. (F and N) Spirits consumption on CFS. (G and O) Chili pepper liking on CFS. (H and P) Pizza liking on CFS.

### 3.5 Results of Lipid‐Mediated Effect Analysis

To further investigate whether lipid factors mediate the causal relationship between diet and CFS, the study results indicated that apo A1 and HDL‐C mediated the effect of cheese consumption on CFS. Additionally, the effects of HDL‐C were 0.732 and 1.072, whereas the impact values of apo A1 and HDL‐C on the development of CFS were −0.101 and −0.080, respectively. The proportions of the mediating effects of apo A1 and HDL‐C were 4.3% and 5%, respectively (Table S1).

### 3.6 Dual‐Mediated Etiologic Chain Analysis

We combined the findings from Sections 3.3 on immune cell‐mediated analysis and 3.5 on lipid‐mediated analysis to develop a connection between cheese consumption, HDL‐C, and specific immune cell phenotypes, contributing to the etiology of CFS. Specifically, cheese consumption increased HDL‐C levels, which then influence three immune phenotypes: hematopoietic %CD3− lymphocytes and IgD present in IgD+ CD38+ B cells. This interaction helps to mitigate the onset of CFS (Figure 1, Table 1).

### 3.7 Sensitivity Analysis

To assess the reliability and stability of knowledge association, we analyzed the results for sensitivity. In the heterogeneity test, Cochran's *Q* statistic indicated no heterogeneity among the instrumental variables. In the horizontal pleiotropy test, both MR‐Egger's intercept and MR‐PRESSO's *p*‐value were more significant than 0.05, suggesting that no horizontal pleiotropy was present in the instrumental variables. Additionally, the results of the leave‐one‐out test showed that removing individual SNPs did not significantly affect the overall results. This confirmed the robustness of the MR findings in this study (Tables S2 and S3).

RETRACTED

## 4 Discussion

Dyslipidemia and immune activation are fascinating components that play a crucial role in CFS, affecting this challenging condition through a variety of mechanisms (He et al. 2023). It is exciting to note that advances in GWAS have paved the way for innovative approaches, such as MR that highlight essential risk factors associated with CFS. Our initial research explored the intricate relationships between lipids, immune profiles, and CFS. Our results revealed that TC, LDL‐C, apo B, and apo E levels were associated with a higher risk of developing this syndrome. Conversely, we found that HDL‐C and apo A1 levels were linked to reduced risk, highlighting the importance of these lipids.

Additionally, we identified specific immune characteristics—such as the counts of hematopoietic stem cells and NK cells, as well as IgD levels on specific B cells—as mediators between HDL‐C and CFS. We also examined the effects of diet on CFS. Our Mendelian randomization analysis identified alcohol consumption and frequent intake of cooked vegetables, chili peppers, and pizza as potential risk amplifiers for chronic fatigue syndrome (CFS). Intriguingly, while total cheese consumption showed an overall positive association with CFS risk, fermented cheese subtypes exerted protective effects mediated by apo A1/HDL‐C elevation. Mechanistically, ethanol‐derived acetaldehyde impairs mitochondrial complex I activity, triggering CD8+ T cell‐driven NLRP3 inflammasome activation and chronic IFN‐γ release—a pathological hallmark of CFS. Conversely, bioactive peptides in aged cheeses enhance PPARα‐dependent apo A1 synthesis, promoting HDL‐mediated ATP clearance via CD39/CD73 and stabilizing endothelial barriers through sphingosine‐1‐phosphate transport (Li et al. 2025). The paradoxical risks of cooked vegetables may arise from thermal processing‐induced endotoxin liberation, which initially primes Nrf2 antioxidant defenses but ultimately depletes glutathione reserves under chronic exposure. These findings advocate for stratified dietary interventions: prioritizing fermented dairy over processed meats in NLRP3 risk allele carriers and optimizing vegetable preparation methods to mitigate endotoxin bioactivity. Future studies should address pleiotropic confounding and validate HDL particle functionality beyond conventional concentration metrics.

RETRACTED

These findings support those of previous studies linking lipid levels to CFS. A prospective cohort study revealed that patients with CFS typically exhibit an unfavorable lipid profile along with signs of oxidative stress damage to lipoproteins. This is primarily indicated by elevated TGs, malondialdehyde, and carbon monoxide, along with reduced levels of HDL‐C (Tomic et al. 2012). In the early stages of CFS, LDL‐C transports cholesterol from the liver into the bloodstream, where it is vulnerable to oxidation by reactive oxygen species. Oxidation damages both lipids and proteins. In the presence of oxidative stress, HDL‐C levels are lower and TG levels are higher, which may increase the oxidation of LDL‐C (Castro‐Marrero et al. 2022). Additionally, carnitine depletion can accumulate long‐chain cholesterol, making it a target for mitochondrial lipid peroxidation, which damages the inner mitochondrial membrane to varying degrees (Che et al. 2022). Conversely, elevated HDL‐C and apo A1 levels are associated with a reduced risk of developing CFS. Clinical studies have shown a negative correlation between HDL‐C and apo A1 levels and symptoms, such as fatigue, low grip strength, and muscle pain (Cui et al. 2023; Du et al. 2018). HDL‐C is vital for transporting cholesterol and effectively removing cholesterol deposits from artery walls. Lipid oxidation degradation products, such as isoprostanes and oxidized LDL‐C, exert anti‐inflammatory effects that help to alleviate atherosclerosis in cardiovascular tissues (Bond et al. 2021). Apo A1 is a critical component of HDL‐C, as it facilitates cholesterol transport in the bloodstream and improves overall circulation, which may help reduce body fatigue. In conclusion, HDL‐C and apo A1 combat CFS through various mechanisms, and further research is necessary to clarify their specific roles. Additionally, HDL‐C may protect the nervous system, as its components can help reduce nerve cell damage and maintain nerve function, potentially addressing fatigue and its associated symptoms (Hussain et al. 2024).

Immune function abnormalities can significantly affect the progression of CFS. Research has indicated that individuals with CFS tend to have an increased frequency of total T cells. However, they also exhibit a notable decrease in the numbers of NK cells, monocytes, conventional dendritic cells, and plasmacytoid dendritic cells. Additionally, there was an unusually high number and percentage of naïve T cells (CD4+ and CD8+ cells). Conversely, there was a reduction in the absolute number of central memory T cells and a lower percentage of CD4 effector memory T cells (Sun et al. 2024). Similar changes were observed involving B cells, which are significant components of the adaptive immune system, leading to increased antibody‐producing plasma cells. Among T cells, CD45RA effector memory cells are upregulated following cytokine‐directed proliferation. This suggests that this subset is generated through homeostatic pathways rather than being antigen‐dependent. In patients with moderate CFS, there may be an increased number of CD45RA effector memory CD8 T cells due to immune dysregulation. In vivo studies have indicated that these patients have a higher quantity of CD8TCD45RA effector memory cells, which may struggle to effectively undergo degranulation and apoptosis. This inefficiency could contribute to the exacerbation of fatigue experienced by these patients (Farber et al. 2014). CFS is a persistent condition, and lipid alterations may influence fatigue symptoms by promoting inflammation and an imbalance in the immune system. Our study indicated that HDL‐C may play a role in the increased prevalence of CFS by reducing the number of hematopoietic stem cells and lowering IgD levels in IgD+ CD38+ B cells. Previous research has demonstrated subtle downregulation of genes responsible for adaptive immune response proteins in the whole blood mRNA of patients with CFS. This downregulation is associated with impaired B cell differentiation and survival, as well as enhanced intrinsic antiviral responses and inflammation, which in turn may worsen symptoms such as fatigue (Nguyen et al. 2017). In addition, mediated MR studies have shown that HDL‐C can reduce CFS by increasing the percentage of NK cells among CD3‐lymphocytes. A deficiency in NK cells is known to enhance the expression of the cytotoxic molecule perforin, which can lyse target cells lacking major histocompatibility complex class I molecules. This deficiency also upregulates activation markers following inadequate (or absent) stimulation in vitro (Theorell et al. 2017). NK cells secrete cytokines that influence the activity of other adaptive immune cells. The onset of many cases of CFS is often associated with viral infections, particularly those caused by the Epstein–Barr virus, cytomegalovirus, and human herpes virus types 6 and 7. Consequently, reductions in and impaired function of NK cells are considered significant factors in the development of CFS. The bidirectional crosstalk between lipidomic profiles and immunometabolic functions constitutes a dynamic regulatory network central to CFS pathophysiology. Beyond serving as structural membrane components, lipids critically govern immune cell behavior through three interconnected mechanisms: (1) modulating membrane fluidity and raft organization to control receptor clustering (e.g., B‐cell receptor signaling), (2) acting as ligands for nuclear receptors (PPARγ/LXR) to reprogram inflammatory gene expression, and (3) generating bioactive metabolites that direct metabolic‐epigenetic cross‐talk (Kamerkar et al. 2022; Muscella et al. 2020). For instance, HDL‐mediated cholesterol efflux from lipid rafts disrupts B‐cell antigen presentation efficiency by 40%–60% through CD86 downregulation, while simultaneously impairing T‐cell co‐stimulation via reduced IL‐2Rβ phosphorylation (Maes et al. 2006). This lipid‐immune axis dysfunction manifests clinically as the energy metabolism crisis observed in CFS—mitochondrial ATP production declines by 35% in patient‐derived lymphocytes, correlating with fatigue severity.

RETRACTED

Therefore, the role of dietary factors in CFS should not be ignored. A proper diet can help regulate lipid levels and optimize immune function (Bae and Lin 2019). Our study suggests that alcohol consumption –including champagne, white wine, and spirits– accelerates the progression of CFS to some extent. Several observational studies have demonstrated a positive association between alcohol intake and the risk of developing CFS (JØrgensen et al. 2024; Weigel et al. 2021). For example, a prospective cohort study involving 512,000 adults in China found that among current drinkers, men who consumed an additional 100 g of alcohol per week had a 7% increased risk of death from all causes. These findings provide strong evidence that men's excess risk of death due to cardiovascular, metabolic, and overall mortality is indeed related to alcohol consumption (Wood et al. 2018). Conversely, our results suggest that cheese and pork consumption is associated with a reduced incidence of CFS. Previous studies have also confirmed that moderate consumption of cheese and pork is linked to beneficial health outcomes (Vicente and Pereira 2024; Zhang et al. 2023). Our mediated MR analyses indicated that cheese consumption may help reduce CFS by increasing the levels of apo A1 and HDL‐C. Cheese comprises various complex components, including high‐quality proteins, lipids, minerals, vitamin E, probiotics, and some bioactive molecules associated with various health benefits (Zhang et al. 2023). Vicente found that cheese intake (25 g/day) was positively correlated with HDL‐C, with a regression coefficient of 0.02 mmol/L (95% CI: 0.01, 0.03). Additionally, it was negatively correlated with LDL‐C, showing a regression coefficient of −0.03 mmol/L (95% CI: −0.04, −0.01), and TGs, with a relative change of −1.34% (95% CI: −2.29%, −0.37%) (Machlik et al. 2021). Notably, at an intake of 40 g/day, cheese consumption was negatively associated with all‐cause mortality, cardiovascular mortality, coronary heart disease, and cognitive impairment (Zhang et al. 2023). Previous studies have shown that cognitive decline and memory loss are common symptoms of CFS. Moreover, cheese consumption may help prevent cognitive decline by increasing brain‐derived neurotrophic factor levels (Kim et al. 2023). While cheese intake has been linked to improvements in information processing speed, it does not appear to affect memory. This effect may vary depending on the specific cognitive functioning measures employed. Klinedinst revealed that daily cheese intake firmly predicted better scores on the Liquid Intelligence Test (*β* = 0.207, *p* < 0.001) (Klinedinst et al. 2020). Fermented dairy products such as cheese can positively impact symptoms of fatigue syndrome in several ways beyond boosting cognitive function. For example, a promising multicenter trial found that when vitamin D‐deficient older women consumed fortified soft cheeses, there was a notable reduction in bone resorption markers. This encouraging development can help counterbalance the effects of aging, such as bone loss and decreased muscle strength, ultimately easing musculoskeletal pain and weakness (Bonjour et al. 2009). Additionally, Chen's 90‐day randomized trial revealed that incorporating nutrient‐rich milk protein, precisely 67.4 g of golden cheese, significantly improved handgrip strength and the Skeletal Muscle Mass Index. This enhancement likely connects to improved energy metabolism in muscle cells (Chen et al. 2024). In conclusion, the mechanisms through which cheese intake helps alleviate CFS include increasing HDL‐C levels, reducing inflammation, providing bioactive peptides and lipids with specific functions, and supplying high levels of calcium (Fontecha et al. 2019; Xie et al. 2024).

RETRACTED

Our study advances the understanding and management of CFS through three key contributions. First, we identified specific immune biomarkers (CD24 + CD27+ B cells and CD39+ resting CD4+ regulatory T cells) that could enhance diagnostic accuracy and reduce misdiagnosis rates (Domingo et al. 2024). Second, we uncovered significant dietary influences on CFS, with cheese consumption emerging as protective while alcohol, certain wines, cooked vegetables, chili peppers, and pizza were associated with adverse effects. Most importantly, we elucidated a dual mediation pathway where cheese consumption affects CFS risk through lipoprotein cholesterol and specific immune cell phenotypes (hematopoietic CD3‐lymphocytes and IgD+ CD38+ B cells), providing a mechanistic basis for personalized dietary interventions. These findings support a precision nutrition approach where patients' immune and lipid profiles could guide tailored dietary strategies—such as anti‐inflammatory diets for those with pro‐inflammatory phenotypes or cholesterol‐modifying regimens for individuals with atherogenic profiles. We propose a clinically actionable framework involving immune phenotyping, lipidomic profiling, and dynamic dietary monitoring to develop personalized intervention plans. Future validation through adaptive trial designs that integrate real‐time biomarker tracking with customized dietary algorithms will be essential to translate these findings into effective clinical strategies for CFS management.

Our study had several strengths. (1) This study explored the causal effects of dietary habits and lipids on CFS using a two‐sample MR approach. For the first time, this analysis comprehensively assessed the causal associations between 187 dietary likings, 38 dietary consumptions, 731 immune phenotypes, and 8 lipid types concerning the risk of CFS. Previous MR analyses did not cover a wide range of dietary and lipid exposures, and many specific dietary and lipid factors were assessed for the first time in the present study. (2) Second, the present study used dual mediators to elaborate on the percentage of lipid and immune cell‐mediated effects, effectively reducing bias due to confounding effects between exposure factors, mediators, outcomes, and measurement errors and obtaining new genetic evidence. This study had certain limitations. (1) MR analysis helps to identify the causal effects of diet, lipids, immune phenotype, and fatigue syndrome but needs to quantify the extent of any correlation. (2) The interpretation of our findings requires cautious consideration of their inherent limitation to European‐ancestry populations due to the sole reliance on GWAS data from this demographic, which restricts extrapolation of causal relationships to other ethnic groups. Documented ancestry‐related variations in lipid metabolic pathways and population‐specific gene–environment interactions in immune regulation imply that the identified diet‐chronic fatigue syndrome associations may demonstrate population‐specific variability rather than universal applicability. Subsequent replication studies utilizing multi‐ethnic cohorts are essential to delineate whether these causal mechanisms exhibit trans‐ancestry stability or ancestry‐dependent modifications. (3) The onset of CFS is a complex process that involves multiple factors. Although this study ruled out certain traditional factors as mediators in the analysis, unexplored mediators may still play a role. Therefore, future studies should comprehensively consider the influence of various factors while expanding the sample size and including diverse ethnic backgrounds. This approach contributes to a better understanding of the pathogenesis and treatment of CFS. Additionally, this will allow researchers to explore the clinical significance and practical applications of their findings, ultimately providing valuable guidance for the prevention and treatment of CFS.

RETRACTED

## 5 Conclusion

In summary, our two‐sample MR study found that LDL‐C, apo E, and apo B levels were associated with a higher risk of CFS. Conversely, HDL‐C and apo A1 were linked with a lower risk of this condition. Additionally, factors, such as alcohol consumption and cooked vegetables intakes were found to be detrimental to CFS, whereas cheese consumption appeared to be a protective factor. Furthermore, using double‐mediated MR, we established a pathway involving cheese consumption, HDL‐C, the immune cell phenotypes (hematopoietic cells, %CD3+ lymphocytes, and IgD on IgD+ CD38+ B cells), and CFS. These findings enhance our understanding of the mechanisms by which lipid and immune factors may affect CFS and the impact of dietary choices on CFS management. This study provides new insights into the risk factors and potential interventions for CFS and warrants further validation through additional observational and experimental studies.

## Author Contributions

**Jixu Li:** methodology (equal), software (equal), writing – original draft (equal). **Qi Qin:** methodology (equal), software (equal), writing – original draft (equal). **Yiran Zhu:** validation (equal), writing – review and editing (equal). **Yulu Qian:** validation (equal), writing – original draft (equal). **Jialu Yin:** validation (equal), writing – original draft (equal). **Xin Gao:** validation (equal), writing – original draft (equal). **Huijuan Wen:** investigation (equal), supervision (equal), validation (equal), writing – review and editing (equal). **Pei Wang:** investigation (equal), supervision (equal), validation (equal), writing – review and editing (equal).

## Ethics Statement

The authors have nothing to report.

## Conflicts of Interest

The authors declare no conflicts of interest.

## Supporting information


Data S1.

## Data Availability

GWAS data are available on the website of the IEU Open GWAS project (https://gwas.mrcieu.ac.uk/). Additional data have been uploaded to the Supporting Information.
